The article "Cell Recognition Using BP Neural Network Edge Computing" was published in 2022. Journal: Contrast Media Mol Imaging.

# Cell Recognition Using BP Neural Network Edge Computing

**DOI:** 10.1155/2022/7355233

**Published:** 2022-07-12

**Authors:** Xiangxi Du, Muyun Liu, Yanhua Sun

**Affiliations:** ^1^School of Mechanical Engineering, Xi'an Jiaotong University, Xian City 710049, China; ^2^Shenzhen Cellauto Automation Co. Ltd., Shenzhen, China; ^3^National Engineering Research Center of Foundational Technologies for CGT Industy, Shenzhen, China

## Abstract

This exploration is to solve the efficiency and accuracy of cell recognition in biological experiments. Neural network technology is applied to the research of cell image recognition. The cell image recognition problem is solved by constructing an image recognition algorithm. First, with an in-depth understanding of computer functions, as a basic intelligent algorithm, the artificial neural network (ANN) is widely used to solve the problem of image recognition. Recently, the backpropagation neural network (BPNN) algorithm has developed into a powerful pattern recognition tool and has been widely used in image edge detection. Then, the structural model of BPNN is introduced in detail. Given the complexity of cell image recognition, an algorithm based on the ANN and BPNN is used to solve this problem. The BPNN algorithm has multiple advantages, such as simple structure, easy hardware implementation, and good learning effect. Next, an image recognition algorithm based on the BPNN is designed and the image recognition process is optimized in combination with edge computing technology to improve the efficiency of algorithm recognition. The experimental results show that compared with the traditional image pattern recognition algorithm, the recognition accuracy of the designed algorithm for cell images is higher than 93.12%, so it has more advantages for processing the cell image algorithm. The results show that the BPNN edge computing can improve the scientific accuracy of cell recognition results, suggesting that edge computing based on the BPNN has a significant practical value for the research and application of cell recognition.

## 1. Introduction

Recently, cell recognition has become a research hotspot in the field of image processing and pattern recognition and has an extensive application prospect in neurology and biology [1]. The artificial neural network (ANN) plays a very effective role in digital image recognition. The main reason is that neural network has good self-learning behavior, good fault tolerance, and efficient classification efficiency [2]. Among them, the backpropagation neural network (BPNN) is an algorithm tool, which can acquire knowledge through learning and make the network model have the ability to solve problems. It is the most widely used algorithm. Recently, edge computing based on the BPNN has also been favored by multiple researchers. Edge computing is an open platform based on network technology, computing, and storage technology at the end, close to the data source to provide the closest end service for data users. The response end of edge computing is close to the service initiator, so it can provide faster network response services to meet the needs of real-time business processing and security and privacy of the supply chain. The BPNN is used to study the edge detection of the digital image. Based on the analysis of target samples and training samples, its powerful self-learning and self-organization abilities are used to accurately locate the image edge [3]. However, the BPNN algorithm still has many shortcomings, and the development of edge computing is still in its infancy. The edge computing based on the BPNN needs to be further improved to achieve the goal of high recognition accuracy, strong antinoise ability, and short running time.

The BPNN algorithm can be divided into forward propagation and error backpropagation. In forward propagation, the sample data are input, then come to the hidden layer through the input layer, and finally, come to the output layer. If there is an error between the actual output result and the expected output result, it is essential to turn to the error backpropagation process. Each layer of nerve cells will continuously adjust its specific connection weight and threshold according to the gradient descent method to minimize the error value and make the actual output result close to the expected output result [4]. The BPNN has the advantages of large-scale parallel, distributed processing, self-organization, and self-learning. It is widely used in multiple fields and has achieved many outstanding results. Compared with the traditional BPNN algorithm, cell recognition research based on BPNN edge computing is proposed; that is, edge computing is used in the learning and training process of the BPNN algorithm. Only Sobel and Laplacian are selected to segment the cell image. It improves the detection accuracy of specific cell image segmentation effects, plays a good auxiliary role in specific cell recognition, and makes the final detection more efficient and accurate.

## 2. Literature Review

Relevant researchers worldwide have conducted extensive research on the application of neural network technology and edge computing technology. Firdaus and Rhee studied the method of edge computing to deal with the increasing system complexity and data storage problems in the intelligent transportation system. Besides, blockchain and smart contracts were proposed to ensure a reliable environment for secure data storage and sharing in the system. Experiments show that the system can defend against system failures with or without symptoms to reach agreement among consensus participants. Moreover, it is found that the use of an incentive mechanism can promote the system's continuous operation [5]. For the production and export of aquaculture, Zhang proposed a yield prediction model based on an optimized BPNN. The results show that the root mean squared error of the model is less than that of the traditional BPNN, and the learning efficiency is higher than that of the traditional BPNN. It shows excellent performance in processing rich historical data and can shorten the modeling time and obtain good prediction results [6]. Hu et al. studied the application of edge computing technology in the analysis of the organic agricultural supply chain. A trust framework was constructed using the blockchain's invariance and the edge computing paradigm to reduce the cost and improve the operation efficiency of the organic agricultural supply chain. A new consensus mechanism was proposed to manage information flow by classifying stakeholders. The evaluation results show that the designed method can significantly improve performance and reduce cost [7].

As for edge computing, people agree that traditional edge computing has multiple disadvantages, such as a small amount of calculation, simple operation, and high noise sensitivity. However, with the rapid development of artificial intelligence and its wide application in the field of image digital processing, the research of edge computing based on the neural network has emerged. Similarly, the BPNN is the most widely used. The BPNN is optimized by using edge computing technology to improve the operation efficiency of the algorithm. Then, the image feature vector is trained by the BPNN algorithm. Finally, the trained samples are used for image segmentation and edge computing. The research shows that the final image edge is accurate and the segmentation effect is good.

## 3. Cell Recognition Algorithm Based on BPNN Combined with Edge Computing

### 3.1. Application of ANN in Image Recognition

The ANN, also known as the connector model, is a system network based on modern neuroscience, biology, and psychology. Specifically, the ANN system is constructed by imitating the structure and function of human brain nerve cells. Therefore, there is no doubt that its development is closely related to the understanding of human brain structure. Moreover, ANN research is based on the simulation and simplification of the biological nervous system, which reflects the basic characteristics of the biological nervous system to a certain extent [8, 9]. The learning and classification process of the ANN is realized by constantly adjusting the connection weight. It shows that the research purpose of the neural network is to explore the mechanism of human brain processing, storing, and searching information, and then explore the possibility of applying this principle to various signal processing. Besides, most neurons in the neural network have mapping relationships, and they are connected by weight coefficients. Because of this large-scale parallel structure, the neural network is completely different from traditional computers and has a high computing speed.

The pattern recognition of neural networks is mainly divided into the learning process and classification process. Specifically, the first step is the learning process. Massive training samples complete the training process of the network. In this process, according to the specific learning rules, the specific connection weight is constantly adjusted to make the output tend to the direction of manual recognition. In this way, it can be considered that the network has learned the specific internal rules. The ANN is composed of multiple interconnected neurons, and its basic processing unit is the artificial neural unit. Therefore, in the same way, artificial neurons only simulate biological neurons' basic structure and function.  Figure 1 is a specific structural model [10]. The algorithm can be applied to image feature recognition based on this structure.

### 3.2. Application of the BPNN Algorithm in Image Recognition

Rumelhart, an American scholar, first proposed the BPNN. The BPNN is a typical feedforward neural network that combines forward and backward error propagation algorithms. It is widely used because of its multiple advantages, and it is the most widely used neural network [11]. Neural network algorithms can learn in fewer samples and express complex functions with fewer parameters, which reduces the difficulty of setting and adjusting model parameters. Therefore, the sample features that can be learned are richer and their simulation is better.  Figure 2 shows the structural model of the BPNN, which is composed of an input layer, hidden layer, and output layer. Each neuron in the input layer is mainly responsible for receiving external signals and transmitting them to the hidden layer. The hidden layer is the main information processing layer in the neural network, which is responsible for information transformation.

According to the change of information demand, the hidden layer can be a single-layer structure or a multilayer structure. After the information is processed by the hidden layer, it will be transmitted to the output layer. Finally, the output layer outputs the information results to complete the complete network forward propagation [12]. When the actual output result is inconsistent with the expected output result, the network system will enter the error backpropagation stage. After the error passes through the output layer, the connection weight of each layer is modified according to the decline of the error gradient. The feedback information is fed back to the output layer. The hidden layer and input layer are carried out step by step. It is the feedback mechanism of the BPNN and the source of the BPNN name.

A BPNN is a repeated process of information forward transmission and error backward transmission. It is the orderly adjustment of connection weights at all levels to realize the learning and training of the neural network. The weight of neurons in any layer of the BPNN can be determined by partial derivative and learning rate. When using the BPNN for calculation, the above steps need to be repeated until the error between the output value and the expected value reaches the allowable range or the maximum number of iterations of the neural network. This process will continue until the error between the network output and the expected output is minimal or infinitely close, and the number of learning time can be set in advance as needed. The output of the last learning training is the final result [13, 14]. Therefore, applying the BPNN to the process of image recognition can effectively learn the characteristics of the image to better identify the target in the image.

### 3.3. Optimized BPNN Algorithm Based on Edge Computing

In the Internet era, the generation of data is going on all the time. Data storage, encryption, transmission, and other processes may be subject to malicious attacks. Besides, there are huge security risks in databases, edge devices, and cloud storage systems, which are very vulnerable to attacks by hackers and Trojan horse software. Once the data are destroyed and polluted, it will cause serious information loss [15]. Compared with traditional cloud computing, edge computing has obvious advantages, as follows:

1. Low delay and high real-time performance: generally, edge devices are far away from the central server and at the boundary of the whole data system. Therefore, it is close to the data source and can process the data at the first time receiving them, and then transmit them to the central server. The advantage of this is to reduce the pressure of the central server, speed up the data transmission time, and improve the operation efficiency of the central server.
2. Reducing power consumption: the data preprocessing of edge devices can share part of the functions of the central server, greatly reduce the operation pressure of the central server and cloud database, and reduce the power consumption of network broadband.
3. Reducing the risk of centralized data storage and improving the fault tolerance rate of the system: the data no longer need to be uploaded to the cloud server for centralized processing. Hence, part of the storage space can be released and the running speed of the system can be improved. When dealing with complex problems, it frees up more space, avoids system locking, improves fault tolerance, and solves the security problem of data storage [16].

One of the basic features of image processing is image edge, which mainly exists among objects or between objects and their background. With edges, specific images can be segmented, so edge detection aims to segment images. The designed method recognizes two edge conditions in cell image recognition: step edge and roof edge. The specific difference between the two is that the gray level of pixels on both sides of the step edge is significantly different, while the gray level on both sides of the roof edge changes from increase to decrease.  Figure 3 shows the comparison.

In addition, the description method of edge detection uses the derivative of the image gray value function, among which the most representative is the Sobel operator based on the derivative and the Laplace operator based on the second derivative [17, 18]. These operators are based on the weighted average of gray value in a certain neighborhood of a pixel in order to approximate the numerical derivative near the pixel in the algorithm. For a two-dimensional image, the derivative of the gradient corresponding to the two-dimensional function *f* (*x*, *y*) is

(1) $$\begin{array}{c} \nabla f\left(x,y\right)=\left[\begin{array}{c} \partial f\left(x,y\right)/\partial x\\ \partial f\left(x,y\right)/\partial y \end{array}\right]. \end{array}$$

When the change of the derivative cannot express the change of the corresponding gray value in the process of image processing, the second derivative is used. Obviously, the second derivative plays a very important role in the process of image processing. The analysis shows that the extreme point of the derivative, that is, the zero point of the second derivative is a step edge, and the gray values of the pixels on both sides are significantly different [19]. Therefore, edge detection can be realized by calculating the derivative and second derivative of image pixels. The second derivative of common differential operator image is as follows:

(2) $$\begin{array}{c} \nabla^{2}f=\frac{\partial^{2}f}{\partial x^{2}}+\frac{\partial^{2}f}{\partial y^{2}}, \end{array}$$

where *∂*^2^*f*/*∂x*^2^=*f*(*i*, *j*+1) − 2*f*(*i*, *j*)+*f*(*i*, *j* − 1) : *∂*^2^*f*/*∂y*^2^=*f*(*i*+1, *j*) − 2*f*(*i*, *j*)+*f*(*i* − 1, *j*) and *i* and *j* are basic vectors. According to the above gradient calculation equations (1) and (2), the gradient of two-dimensional image *f* (*x*, *y*) at each pixel can be obtained. Then, the pixel can be judged as the edge point according to the obtained pixel gradient [20].

The typical BPNN model includes three levels: input layer, hidden layer, and output layer. If *i*, *j*(*k*), and *θ*_*j*_ are the number of neurons in input, output, and hidden layer or the threshold of neurons, respectively, *w*_*ij*_ is the weight of neurons from input layer to hidden layer.

The calculation equation of the hidden layer is as follows:

(3) $$\begin{array}{c} y_{j}=f\left(\sum_{i=0}^{n}w_{ij}x_{i}-\theta_{j}\right). \end{array}$$

The calculation equation of the output layer is as follows:

(4) $$\begin{array}{c} z_{k}=f\left(\sum_{j=1}^{h}w_{jk}y_{j}-\theta_{jk}\right). \end{array}$$

The error equation of the BPNN algorithm is as follows:

(5) $$\begin{array}{c} E_{r}=\frac{1}{2}{\left\|t_{r}-z_{r}\right\|}^{2}=\frac{1}{2}\sum_{k=1}^{m}{\left(t_{rk}-z_{rk}\right)}^{2}. \end{array}$$

The iterative equation of input layer and hidden layer is as follows:

(6) $$\begin{array}{c} w_{jk}\left(s+1\right)=w_{jk}\left(s\right)+\eta \sum_{r=1}^{N}\delta_{j}x_{i}, \end{array}$$

where *s* is the number of iterations and *δ*_*j*_=*f*′(*u*_*rj*_)∑_*k*=1_^*m*^*δ*_*k*_*w*_*jk*_.

The above description shows that, unlike the activation function of the hidden layer and output layer of BPNN, the sigmoid function is mainly used for edge detection. Its learning process is mainly concentrated in the hidden layer [21, 22]. The main reason for choosing this function as a function of hidden layers is to avoid the saturation of hidden layers. Since the output layer outputs the edge or edge pixel value, and the method to obtain the value is to modify the connection weight along the gradient, the output result is generally the maximum or minimum value.

Besides, to improve the learning efficiency of the network, the Purelin linear function is selected as the activation function of the output layer. The edge computing of the hidden layer of the BPNN is equivalent to the modification of the template coefficient of each operator. The result of the output layer is equivalent to the adjustment of the weight of each operator. The purpose is to achieve the final output result that is infinitely close to the expected value [23]. The cell types involved mainly include red blood cells, white blood cells, and epithelial cells. In the collected cell image dataset, the number of white blood cell images is 138, the number of red blood cell images is 169, and the number of epithelial cell images is 241. Then, the known characteristic signals are used to train the BPNN algorithm.  Table 1 shows the setting of BPNN parameters used.

## 4. Model Test and Analysis

### 4.1. Effect Analysis of Edge Computing

The Sobel operator contains two groups of 3*∗*3 matrices: horizontal and vertical templates. By plane convolution with the image, the approximate values of horizontal and vertical brightness difference can be obtained, respectively. The Laplace operator is a second-order differential operator defined as gradient ∇*f* and divergence ∇*f*′. The second derivative of the image is calculated. The image is two-dimensional, so there is no need to calculate the horizontal and vertical derivatives separately, and then add them. The Sobel operator and Laplace operator are selected to segment the cell image, enhance the region of gray mutation in the image, and weaken the slow-changing region of gray. Two algorithms are used to process epithelial cells.  Figure 4 shows the specific effect.

Figure 4 shows that each operator has its own characteristics in image segmentation. The Laplace operator has high accuracy in image edge detection. However, when there is more noise in the image, the detection accuracy decreases significantly. Besides, the image edge has not only position information but also direction information. However, the Laplace operator can only obtain one aspect of location information. The Sobel operator can smooth and suppress noise, but the actual edge is also smoothed and the detection effect is suppressed, resulting in the decline of detection accuracy. In the groove, the Sobel operator is more suitable for oblique edge detection and the Laplace operator is more suitable for horizontal and vertical edge detection.

### 4.2. Analysis of Network Training Results

In the process of implementing the BPNN, the training process of the BPNN is the most critical. The key of cell recognition is to use the extracted cell features combined with specific network training to carry out the final cell recognition and classification and obtain the recognition results. In order to improve the learning efficiency of the BPNN, edge computing based on the BPNN is used in the hidden layer training process. According to the known collected cell images, the main features are extracted.  Table 2 shows the results. According to the known information, the number of input neurons of the BPNN is 6 and the expected number of output neurons is 3. Then, the BPNN algorithm is trained.

In the BPNN, after the signal from the input layer is received, it reaches the output layer through the hidden layer, and the final result is output. It also experiences a continuous error reduction process. After BPNN algorithm training (the number of hidden layer neurons *S*1 = 15), the output result is shown in Figure 5.

Figure 5 shows that after continuous adjustment, the error of the BPNN output is very close to the expected output. Moreover, the smaller the error between the actual output and the expected result is, the longer the online learning training time is, and the more the training time is. Figure 5 shows the training results.

### 4.3. Analysis of Cell Recognition Results Based on BPNN Combined with Edge Computing

The final recognition result of the BPNN is compared with the actual number of cells to verify the ability of the designed algorithm to deal with the problem.  Table 3 shows the results.

Table 3 displays that the BPNN algorithm can realize the recognition of specific cell types and numbers. The experimental results show that the actual number of white blood cells is 122 and the number of network recognition is 120. There are only two differences, and the accuracy is as high as 98.36%. The actual number of red blood cells is 146, the number of network recognition is 138, and the accuracy rate is 94.52%. The actual number of epithelial cells is 189, and the number of network recognition is 176, with an accuracy of 93.12%. It can be concluded that in BPNN recognition, the recognition effect of white blood cells is the best and that of epithelial cells is the worst.

## 5. Conclusion

Cell recognition is conducted based on BPNN edge computing. This exploration discusses the BPNN structure model and the edge computing process, respectively. Finally, the practical application of BPNN edge computing in cell recognition is discussed, and the following results are obtained. In the process of BPNN recognition, the influence of parameter setting cannot be underestimated. The results show that using the initial weight is a good method in this process because randomly selecting the smallest value will ensure that the nonlinear function is more sensitive than other values in the initial weight. In the training process of the BPNN, the nonlinear mapping relationship between the input layer and output layer can effectively adjust and correct the weight between different levels. When the optimal connection weight between layers is obtained through the continuous iteration of network training, the error between the actual output and the expected output *t* is minimized to obtain the final output value.

The Laplace operator has high accuracy in image edge detection, but the effect of noise suppression is relatively poor. The Sobel operator has a stable noise suppression effect, but the detection accuracy is low. Besides, the cell recognition results based on BPNN edge computing are not different from the actual cell type and number, and the recognition results are accurate, indicating that the effect of BPNN edge computing is very good. However, the edge computing process based on the BPNN is still insufficient in the current research. Further improvement measures can be put forward in terms of sample selection or e-learning strategies. Therefore, there are still many key and difficult problems for many researchers to solve in edge computing based on neural networks.

## Figures and Tables

**Figure 1:** Neuron structure model.

**Figure 2:** BPNN model.

**Figure 3:** Image edge classification: (a) step edge and (b) roof edge.

**Figure 4:** (a) Cell original gray image. (b) Sobel operator segmentation effect. (c) Laplacian operator segmentation effect.

**Figure 5:** Cell recognition training results (*S*1 = 15). The horizontal line is the expected error value.

**Table 1:** BPNN parameter settings.

Parameter	Value
Learning rate	0.3
Maximum training times	100
Accuracy required for training	0
Minimum gradient requirements	1.12E-10
Momentum factor	0.9
The activation function of the output layer	Purelin linear function
Number of network layers	4
Weight change increment	1.2
Reduction of weight change	0.5
Initial weight change	0.07
Loss function	Quadratic mean square function
Activation function	Sigmoid function

**Table 2:** Cell characteristic parameters.

Serial number	Circumference	Area	Roundness	Equivalent diameter	Length	Width
1	39.52	128.00	1.37	12.17	12	13
2	36.32	109.00	1.39	11.78	12	12
3	40.00	132.00	1.45	12.99	13	13
4	39.80	123.00	1.48	12.55	14	12
5	43.20	133.00	1.60	13.05	13	13
6	38.32	118.00	1.46	12.22	13	12
7	36.99	117.00	1.35	12.22	12	12
8	40.38	124.00	1.55	12.55	13	11
9	36.95	109.00	1.43	11.77	13	10
10	38.92	124.00	1.37	12.55	13	11
11	38.99	126.00	1.36	12.65	14	12
12	38.97	125.00	1.39	12.62	13	13
13	38.33	122.00	1.39	12.51	13	11
14	41.81	130.00	1.55	12.88	14	12
15	40.39	131.00	1.44	12.93	13	13
16	42.63	148.00	1.42	13.74	15	13
17	42.05	142.00	1.44	13.46	13	13
18	41.81	138.00	1.44	13.25	13	13

**Table 3:** Cell recognition results.

	Actual number of cells	Cell number recognized by network	Recognition accuracy (%)
White blood cells	122	120	98.36
Red blood cells	146	138	94.52
Epithelial cells	189	176	93.12

## Data Availability

The data used to support the findings of this study are included within the article.
